# Bacteriological Profile and Antimicrobial Susceptibility Patterns of Bacteria Isolated from Pus/Wound Swab Samples from Children Attending a Tertiary Care Hospital in Kathmandu, Nepal

**DOI:** 10.1155/2017/2529085

**Published:** 2017-03-06

**Authors:** Salu Rai, Uday Narayan Yadav, Narayan Dutt Pant, Jaya Krishna Yakha, Prem Prasad Tripathi, Asia Poudel, Binod Lekhak

**Affiliations:** ^1^Department of Microbiology, Goldengate International College, Kathmandu, Nepal; ^2^Forum for Health Research and Development, Dharan, Nepal; ^3^Department of Microbiology, Grande International Hospital, Kathmandu, Nepal; ^4^Central Campus of Technology, Hattisar, Dharan, Nepal; ^5^Department of Microbiology, Kanti Children's Hospital, Kathmandu, Nepal

## Abstract

In Nepal, little is known about the microbiological profile of wound infections in children and their antimicrobial susceptibility patterns. Total of 450 pus/wound swab samples collected were cultured using standard microbiological techniques and the colonies grown were identified with the help of biochemical tests. The antimicrobial susceptibility testing was performed by Kirby-Bauer disc diffusion technique. Methicillin-resistant* Staphylococcus aureus* isolates were detected by using cefoxitin disc and confirmed by determining minimum inhibitory concentrations (MIC) of oxacillin. 264 (59%) samples were culture positive. The highest incidence of bacterial infections was noted in the age group of less than 1 year (76%). Out of 264 growth positive samples, Gram-positive bacteria were isolated from 162 (61%) samples and Gram-negative bacteria were found in 102 (39%) samples.* Staphylococcus aureus* (99%) was the predominant Gram-positive bacteria isolated and* Pseudomonas aeruginosa* (44%) was predominant Gram-negative bacteria. About 19% of* S. aureus* isolates were found to be methicillin-resistant MIC of oxacillin ranging from 4 *μ*g/mL to 128 *μ*g/mL. Among the children of Nepal, those of age less than 1 year were at higher risk of wound infections by bacteria.* Staphylococcus aureus* followed by* Pseudomonas aeruginosa* were the most common bacteria causing wound infections in children.

## 1. Introduction

Injuries among children are major public health problems caused by falls, burns, and road traffic accidents [1]. These various injuries result in development of wounds which drag the patients to the health care facilities. Bacterial infections are serious problems to the successful treatment of the wounds resulting in complications sometimes leading to fatal sepsis. Over 95% of all injury-associated deaths among children occur in low-income and middle-income countries [2].

The common bacterial pathogens responsible for wound infections are* Staphylococcus aureus*,* Pseudomonas aeruginosa*, and bacteria belonging to family Enterobacteriaceae [3].

Since the emergence of methicillin-resistant* Staphylococcus aureus* (MRSA) in 1960, there have been reports of increasing rate of infection by MRSA and this superbug has established itself as the common cause of nosocomial as well as community acquired infections [4]. Further, many reports have shown the increasing rates of infections in children by MRSA [5]. In Nepal, many studies have been conducted to determine the rates of infections caused by MRSA among adults [6], but only limited data are available regarding the prevalence of MRSA among the strains of* S. aureus* isolated from children. Further, from literature review, we concluded that no studies have been conducted to determine the bacteriological profile of wound infections among children and their antimicrobial susceptibility patterns. Children have weak immune system, because of that they are prone to serious infections and timely proper treatment is very necessary. In addition, if the local antimicrobial susceptibility data are not available, the chances of haphazard use of antibiotics will be high. As a result, the rate of drug resistance will increase causing a serious problem. So, in this study, we determined the bacteriological profile of wound infections among children and their antimicrobial susceptibility patterns. Further, we also studied the incidence of methicillin-resistant* Staphylococcus aureus* in causing wound infections among children.

## 2. Methods

### 2.1. Study Design

A cross-sectional study was conducted using total of 450 pus/wound swab samples collected from the children attending Kanti Children's Hospital, Kathmandu, Nepal, from September 2012 to May 2013. The samples were collected from the patients who were admitted to the hospital after surgeries or major injuries and had signs of wound infections. The wounds of the injured patients were cleaned with antiseptic solutions before admitting them to the hospital. So, the patients might have got infections in hospital as the signs of infections were seen after the patients had been admitted.

### 2.2. Isolation, Identification, and Antimicrobial Susceptibility Testing

The samples were subjected to bacteriological culture following standard microbiological techniques [7]. The colonies grown were identified with the help of colony morphology, Gram's staining, and biochemical tests [8]. The antimicrobial susceptibility testing was performed by modified Kirby-Bauer disc diffusion technique following clinical and laboratory standards institute guidelines [9].

### 2.3. Detection of MRSA and Determination of Minimum Inhibitory Concentrations of Oxacillin for Strains of MRSA

MRSA isolates were detected by using cefoxitin disc (30 *μ*g) [9]. Minimum inhibitory concentrations of oxacillin for strains of MRSA (screened by cefoxitin disc diffusion method) were determined by agar dilution method [9, 10].

### 2.4. Quality Control

For quality control,* S. aureus* (ATCC 25923) and* E. coli* (ATCC 25922) were used.

### 2.5. Data Analysis

The data were analyzed by using statistical package for the social sciences version 16.00. *P* value < 0.05 was considered as statistically significant.

## 3. Results

### 3.1. Age-Wise Distribution of Wound Infections

Out of total 450 pus/wound swab samples processed, 264 (59%) were culture positive. The highest incidence of bacterial infections was noted in the age group of less than 1 year (76%), followed by the age group of 1–5 years (69%), 5–10 years (58%), and 10–15 years (33%).

### 3.2. Bacteriological Profile of Wound Infections

Out of 264 growth positive samples, Gram-positive bacteria were isolated from 162 (61%) samples and Gram-negative bacteria were found in 102 (39%) samples. Among Gram-positive isolates, 160 (99%) were* Staphylococcus aureus* and 2 (1%) were* Streptococcus pyogenes*. Similarly, among Gram-negative isolates, the most prevalent bacteria isolated were* Pseudomonas aeruginosa,* 45 (44%), followed by* Klebsiella pneumoniae*, 28 (27%);* Escherichia coli*, 13 (13%),* Acinetobacter* spp., 7 (7%);* Citrobacter koseri*, 4 (4%);* Proteus mirabilis*, 3 (3%); and* Citrobacter freundii*, 2 (2%) (Table 1). The bacteriological profile of wound infections among children was similar to that of adults.

### 3.3. Antibiotic Susceptibility Patterns of* S. aureus*

Highest rate of susceptibility was seen toward cefoxitin (81%) followed by gentamicin (76%). 31 (19%) isolates were resistant to cefoxitin and were screened as methicillin-resistant* S. aureus* (Table 2).

### 3.4. Minimum Inhibitory Concentrations of Oxacillin for MRSA Screened by Cefoxitin Disc Diffusion Method

All the 31 MRSA isolates screened by cefoxitin disc diffusion method had minimum inhibitory concentrations of oxacillin ≥ 4 *μ*g/mL. The MIC values ranged from 4 *μ*g/mL to 128 *μ*g/mL.

### 3.5. Antibiotic Susceptibility Patterns of Gram-Negative Bacilli

Highest rate of susceptibility was seen toward amikacin (49%), followed by ciprofloxacin (44%) (Table 3).

### 3.6. Antibiotic Susceptibility Patterns of* Pseudomonas aeruginosa*

Highest rate of susceptibility was seen toward ciprofloxacin (51%), followed by tobramycin (44%) (Table 4).

### 3.7. Antibiotic Susceptibility Patterns of* K. pneumoniae*

Highest rate of susceptibility was seen toward cefixime (57%) (Table 5).

## 4. Discussion

Wound infection is one of the most common and serious complications among the hospital acquired infections [11–13]. Wound infection can increase the length of hospital stay and accounts for the mortality rate up to 70–80% [12, 13]. The growth positivity reported by Bhatta and Lakhey (60%) was similar to our finding [14]. However, lower rate was reported by Shrestha and Basnet (50%) [15].

The result obtained showed the slightly decreasing trend in rates of wound infections with increase in age. And highest rate of wound infection was among the children below 1 year of age. Our finding was in accordance with the findings by Kai-Yang et al. [16] and Önen et al. [17]. Due to the weak immune system of the younger children, they are more susceptible to infections.

As in our study, Bhatta and Lakhey [14], Shrestha and Basnet [15], and Garba et al. [18] also reported the* S. aureus* to be the most prevalent bacteria isolated from the cases of wound infections. In hospital the sources of* S. aureus* may be the inanimate objects, health care workers, and other patients. Further, due to presence of the* S. aureus* as normal flora of human body, the endogenous infections are also possible.

The relatively higher resistance of the bacteria isolated from the children to the commonly used antibiotics is a matter of great concern. The prevalence of MRSA reported in our study was in accordance with that reported by Subedi and Brahmadathan (15.4%) [19]. However, higher rates were reported by Kshetry et al. (37.6%) [6], Sanjana et al. (39.6%) [20], Dibah et al. (46.3%) [21], and Tiwari et al. (69.1%) [22]. In a recent study from Nepal, Adhikari et al. also reported higher rate of MRSA in comparison to our study [23]. The difference in the rates of isolation of MRSA in different studies might be due to the difference in the level of irrational antibiotic use, level of hygienic condition maintained in different hospitals, and effective implementation of hand hygiene program. But the high rate of isolation of MRSA from the children indicates a serious problem. The treatment of infection caused by MRSA may require the use of reserve drug, vancomycin. The use of vancomycin in children may cause the emergence of the vancomycin-resistant Gram-positive bacteria, leaving little or no option for the treatment of serious infections caused by those superbugs.

## 5. Limitations of the Study

Because of resource constraints, we were unable to use molecular level analysis to confirm our results. Further, multicenter study including larger numbers of samples would have generated more significant results.

## 6. Conclusions

Among the children of Nepal, those of age less than 1 year were at higher risk of wound infections by bacteria and there was a decreasing trend in rates of wound infections with increase in age.* Staphylococcus aureus* followed by* Pseudomonas aeruginosa* were the most common bacteria causing wound infections in children, which are also the predominant pathogens causing wound infections in adults.

## Figures and Tables

**Table 1:** Results of biochemical tests of different bacteria isolated in our study.

Yellow colony on mannitol salt agar, Gram-positive cocci, catalase positive, slide and tube coagulase positive, gelatin hydrolysis positive, beta-hemolysis in blood agar, methyl red test and Voges-Proskauer test positive, nitrate reduction positive	*S. aureus*

Gram-positive cocci, catalase negative, beta-hemolysis in blood agar, bacitracin sensitive, bile-esculin test negative, L-pyrrolidonyl-*β*-naphthylamide (PYR) test positive	*S. pyogenes*

Gram-negative bacilli, oxidase positive, catalase positive, greenish yellow colonies on nutrient agar, citrate positive, motile, indole negative, urease negative, lactose non-fermenting, hydrogen sulphide negative, gas negative	*P. aeruginosa*

Gram-negative bacilli, catalase positive, oxidase negative, mucoid colony, nonmotile, urease positive, citrate positive, indole negative, lactose fermenting, gas positive, hydrogen sulphide negative	*K. pneumoniae*

Gram-negative bacilli, catalase positive, oxidase negative, motile, urease negative, citrate negative, indole positive, lactose fermenting, gas positive, hydrogen sulphide negative	*E. coli*

Gram-negative bacilli, catalase positive, oxidase negative, citrate positive, lactose non-fermenting, indole negative, nonmotile, gas negative, hydrogen sulphide negative	*Acinetobacter* spp.

Gram-negative bacilli, oxidase negative, catalase positive, lactose fermenting, indole negative, motile, urease differential, hydrogen sulphide positive, gas positive, citrate positive	*C. freundii*

Gram-negative bacilli, oxidase negative, catalase positive, lactose non-fermenting, indole positive, motile, urease differential, hydrogen sulphide negative, gas positive, citrate positive	*C. koseri*

Gram-negative bacilli, oxidase negative, catalase positive, lactose non-fermenting, indole negative, motile, urease positive, hydrogen sulphide positive, gas positive, citrate positive	*P. mirabilis*

**Table 2:** Antibiotic susceptibility patterns of *S. aureus*.

Antibiotics	Sensitive (%)
Cefoxitin	129 (81%)
Amoxicillin	46 (29%)
Gentamicin	122 (76%)
Cefotaxime	100 (63%)
Erythromycin	115 (72%)
Ciprofloxacin	101 (63%)
Cotrimoxazole	89 (56%)

**Table 3:** Antibiotic susceptibility patterns of Gram-negative bacilli.

Antibiotics	Sensitive (%)
Amikacin	50 (49%)
Ciprofloxacin	45 (44%)
Ofloxacin	35 (34%)
Ceftazidime	34 (33%)
Cotrimoxazole	36 (35%)
Cefixime	42 (41%)

**Table 4:** Antibiotic susceptibility patterns of *Pseudomonas aeruginosa* (*n* = 45).

Antibiotics	Sensitive (%)
Amikacin	13 (29%)
Ciprofloxacin	23 (51%)
Ofloxacin	9 (20%)
Ceftazidime	13 (29%)
Cotrimoxazole	14 (31%)
Cefixime	16 (36%)
Tobramycin	20 (44%)

**Table 5:** Antibiotic susceptibility patterns of *K. pneumoniae *(*n* = 28).

Antibiotics	Sensitive (%)
Amikacin	10 (36%)
Ciprofloxacin	11 (39%)
Ofloxacin	11 (39%)
Ceftazidime	8 (29%)
Cotrimoxazole	10 (36%)
Cefixime	16 (57%)

## Abbreviations

CLSI: Clinical and Laboratory Standards Institute
ATCC: American Type Culture Collection
MRSA: Methicillin-resistant* Staphylococcus aureus*
MIC: Minimum inhibitory concentration.
